# Analysis of Risk Factors and Surgical Strategy of Knee Traumatic Arthritis after Internal Plate Fixation in the Treatment of Tibial Plateau Fracture

**DOI:** 10.1155/2022/9146227

**Published:** 2022-09-05

**Authors:** Xingming Jin, Dengying Li, Lei Yang, Fuyuan Han, Pinwu Jia

**Affiliations:** Department of Ortheopaedies, Central Hospital of Jinchang City, Gansu Province 737100, China

## Abstract

**Objective:**

To explore the risk factors and surgical strategies of knee traumatic arthritis after internal plate fixation in the treatment of tibial plateau fracture.

**Methods:**

A total of 300 patients with tibial plateau fractures treated with internal plate fixation in our hospital from January 2019 to April 2021 were retrospectively analyzed. According to whether secondary knee traumatic arthritis occurred after operation, they were divided into control group and research group. The control group was nonsecondary knee traumatic arthritis (*n* = 231), and the research group was secondary knee traumatic arthritis (*n* = 69). Univariate and multivariate logistic regression analysis was used in this research.

**Results:**

There were significant differences in fracture classification, injury method, osteoporosis, and the time from injury to operation between the two groups, and there are statistically significant differences between groups (*P* < 0.05). Fracture type, injury method, osteoporosis, and time from injury to operation were the influencing factors of tibial internal fixation, and there are statistically significant differences between groups (*P* < 0.05). Platform fracture was an independent risk factor for postoperative knee joint traumatic arthritis, and there are statistically significant differences between groups (*P* < 0.05). The HSS scores of both groups increased after operation, and there are statistically significant differences between groups (*P* < 0.05). No loosening of the prosthesis was found in all 69 patients with postoperative X-ray examination.

**Conclusion:**

Fracture classification, injury mode, osteoporosis, and time from injury to operation are independent risk factors for knee traumatic arthritis in the treatment of tibial plateau fractures with internal plate fixation, incidence of knee trauma.

## 1. Introduction

Tibial plateau fractures are the most common fracture in knee trauma, accounting for 8 percent of fractures in the elderly [1]. Tibial plateau fractures are mostly caused by high-energy injuries, accounting for about 1% of systemic fractures. The incidence of posterolateral fractures is relatively low, accounting for 8%. Tibial plateau fracture is easy to be accompanied by different degrees of soft tissue injuries such as cruciate ligament and collateral ligament, which is relatively difficult to deal with [2]. Surgical methods are often used to treat tibial plateau fractures in order to restore the painless knee joint with stable structure, good line of force and good movement as far as possible. As most of the tibial plateau fractures are high-energy injuries in different directions, the injury mechanism is very complex, and clinical surgical treatment is difficult [3]. Complex tibial plateau fractures are often accompanied by severe soft tissue injuries, which are difficult to treat in clinic. Improper treatment of soft tissue injuries associated with tibial plateau fractures can seriously affect the normal function of the knee joint, leading to traumatic arthritis and knee valgus deformity [4].

With the aging of population, the incidence of tibial fractures has risen sharply. The tibial plateau is one of the important load-bearing joints in the human body, and it is usually an intra-articular fracture [5]. With the development and progress of minimally invasive technology, minimally invasive methods have also been introduced into internal fixation technology. Minimally invasive percutaneous plate osteosynthesis (MIPPO) does not need to rely on the adhesion between the plate and the fracture end. Keeping a certain distance between the two can significantly reduce soft tissue damage and provide sufficient blood to the fracture end to the greatest extent. It can promote the healing of fracture ends [6]. Foreign scholars have reported that the use of MIPPO technology combined with L-type and T-type plates in the treatment of patients of different ages has a satisfactory clinical effect and can minimize the pain of patients, which is beneficial to early rehabilitation exercise [7]. However, for elderly patients with degenerative joint disease, intra-articular fractures will be more serious and the clinical effect is not good. Minimally invasive internal fixation systems are not perfect, and there is a risk of secondary traumatic knee arthritis after surgery. In view of this, this study would investigate the risk factors affecting the secondary traumatic arthritis of the knee after the treatment of tibial plateau fractures with internal plate fixation.

## 2. Materials and Methods

### 2.1. General Information

A total of 300 patients with tibial plateau fracture treated by internal plate fixation in our hospital from January 2019 to April 2021 were retrospectively analyzed. According to whether secondary knee traumatic arthritis occurred after operation, they were divided into control group and research group. The control group was nonsecondary knee traumatic arthritis (*n* = 231), and the research group was secondary knee traumatic arthritis (*n* = 69). The general data of the two groups of patients were shown in Table 1. This study was approved by the Medical Ethics Association of our hospital.

Diagnostic criteria of tibial plateau fracture: the patient had a history of trauma such as falling. And there were symptoms such as pain, swelling, and limitation of movement of the affected knee joint. Combined with CT, X-ray, and other imaging examination, the diagnosis was in line with the relevant diagnostic criteria of tibial plateau fracture [8].

Selection criteria: (1) all the patients were simple tibial plateau fractures and were voluntarily treated with internal plate fixation; (2) freshly closed single limb fractures without vascular and nerve injury; (3) postoperative rehabilitation exercise according to the doctor's advice, regular reexamination, and complete follow-up.

Exclusion criteria: (1) patients with open fracture, pathological fracture, and old fracture; (2) complications such as osteofascial compartment syndrome and deep venous thrombosis of lower extremities; (3) patients with dysfunction of the affected limb, such as myasthenia gravis and paraplegia; (4) patients who could not cooperate with functional exercise and follow-up after operation; (5) patients with serious medical diseases, poor physique, and mental illness.

### 2.2. Operation Methods

All patients were treated by the same surgical team and were treated with continuous epidural anesthesia before operation. The healthy side was taken from the recumbent position, and the epidural catheter was placed in L1-2 or L2-3 lumbar intervertebral space. After seeing the reflux of cerebrospinal fluid, the anesthetic was injected slowly, and the anesthetic was 5 mg. The patient was changed to a supine position, and the procedure was performed under the control of a balloon tourniquet. For patients with displaced fractures of type I according to Schatzker's classification [9], cannulated compression screw fixation was performed. Patients with type II and type III fractures were treated with lateral incision, patients with type IV fractures were treated with medial knee incision or a straight incision close to the midline, and type V fractures were treated with a lateral incision. Type VI fracture patients chose a straight incision close to the midline. Cut open the joint capsule and coronary ligament, check the injury of meniscus and ligament, show the tibial plateau from below the meniscus, retain the meniscus as far as possible during the operation, and remove the seriously injured meniscus. Expose the fracture end, observe the collapse of the platform, pry up the fracture block in the proximal tibia for the collapsed fracture of the articular surface, repair the articular surface, fix it temporarily, and insert the autogenous iliac bone into the defect of the proximal tibia to repair the bone defect and ligament repair. After satisfactory reduction by C-arm X-ray machine, the cancellous bone screws and anatomical plates selected in advance were fixed. Suture the coronal ligament and repair the injured meniscus and ligament. The ligament injury with avulsion bone mass was fixed in the first stage during the operation. For the patients with injury of the solid part of cruciate ligament, the primary repair or reconstruction could not be done during the operation, but the second-stage ligament reconstruction can be done. Negative pressure drainage and pressure bandaging were performed after operation.

### 2.3. Observation Index

#### 2.3.1. Incidence of Traumatic Knee Arthritis

After the completion of the operation, 300 patients were followed up for 1 year, and the incidence of traumatic arthritis within 1 year after operation was calculated. Diagnostic criteria of knee traumatic arthritis [10]: (1) there was a history of trauma (surgery is also a history of external injury); (2) the early lesion was characterized by joint pain and discomfort, especially stiffness after exercise, which was improved after proper exercise massage, but did not overwork; (3) when the disease progresses to the later stage, there might be severe symptoms such as limitation of movement, repeated swelling of the joint, persistent pain and gradual aggravation, joint deformity, and effusion; (4) X-ray examination showed the narrowing of joint space and the formation of bone spur at the edge of subchondral articular surface sclerosis. For patients with severe condition, it could be characterized by irregular articular surface, bone end deformation, and loose body in the joint.

#### 2.3.2. General Information

The age, sex, type of plate, meniscus injury, ligament injury, fracture classification, osteoporosis, mode of injury, time from injury to operation, weight bearing time after operation (5 kg) and whether to remove internal fixation were recorded in the two groups. (1) Determination of meniscus injury [11]: by asking the patient's symptoms, combined with freehand examination, imaging examination, and arthroscopy. If the patient has the symptoms of joint swelling and limitation of movement, the joint, joint space, and meniscus feel tenderness during physical examination, MRI examination shows meniscus grade III signal changes; combined with arthroscopy, the existence of meniscus injury can be comprehensively determined. (2) Determination of ligament injury [12]: ligament injury can be divided into two types: collateral ligament injury and cruciate ligament injury. (3) Determination of osteoporosis [13]: the existence of osteoporosis was determined by whole body bone mineral density (BMD). If the bone mineral density was less than-2.5, it can be diagnosed as osteoporosis. (4) Determination of high-energy and low-energy injuries [14]: high-energy injuries referred to complex injuries caused by direct impact injury and changes in limb position at the same time. In addition to more combined injuries, limb fractures have a wide range of fractures and serious comminution. Local tissue was severely injured, generally accompanied by obvious soft tissue damage. The low-energy injury referred to the direct impact injury, the range of limb fracture was small, and the degree of local tissue trauma was low.

#### 2.3.3. Analysis of Risk Factors of Postoperative Knee Traumatic Arthritis

Differences in the incidence of postoperative knee traumatic arthritis in patients with different clinical characteristics were included in a multivariate logistic regression model.

#### 2.3.4. Surgical Effect

The knee function and acetabular bone healing of patients with secondary knee traumatic arthritis after total knee arthroplasty and total knee joint surface placement were recorded. The improvement of knee joint function was evaluated by HSS score [15]. The total score of the scoring system was 100. The score was proportional to the function of hip joint.

### 2.4. Statistical Analysis

SPSS 22.0 statistical software was used to analyze the data. Measurement data are expressed as mean ± standard deviation (*x* ± *s*) using *t*-test or analysis of variance; those that do not conform to the normal distribution are represented by the median (quartile interval). Rank sum test was used, counting data was expressed by the number of cases and percentage, *χ*^2^ test was used, and binary logistic regression analysis was used to screen the influencing factors of knee osteoarthritis. The difference was statistically significant, and the difference was statistically significant, and there are statistically significant differences between groups (*P* < 0.05).

## 3. Results

### 3.1. Incidence of Secondary Knee Traumatic Arthritis after Operation

The incidence of knee traumatic arthritis after internal plate fixation in the treatment of tibial plateau fracture: 69 cases of knee traumatic arthritis occurred in 300 patients with tibial plateau fracture after internal plate fixation with an incidence of 23%. All results are shown in Figure 1.

### 3.2. Monofactor Analysis of Knee Traumatic Arthritis after Internal Plate Fixation in the Treatment of Tibial Plateau Fracture

There was no significant difference in age, sex, type of plate, meniscus injury, cruciate ligament injury, collateral ligament injury, weight bearing time, and internal fixation between the control group and the research group (*P* > 0.05). There were significant differences in fracture classification, mode of injury, osteoporosis, and time from injury to operation between the two groups, and there are statistically significant differences between groups (*P* < 0.05). All the data results are shown in Table 1.

### 3.3. Logistic Regression Analysis of Multiple Factors Affecting Knee Traumatic Arthritis after Internal Plate Fixation in the Treatment of Tibial Plateau Fracture

Internal plate fixation in the treatment of tibial plateau fracture after knee traumatic arthritis as a constant, fracture classification, mode of injury, osteoporosis, and injury to operation time as dependent variables are shown in Table 2. Multivariate logistic regression analysis showed that fracture classification, injury method, osteoporosis, and the time from injury to operation were the factors that led to the treatment of tibia with internal plate fixation. The independent risk factors of postoperative knee traumatic arthritis after platform fracture surgery were statistically different, and there are statistically significant differences between groups (*P* < 0.05). All results are shown in Table 3.

### 3.4. Curative Effect and Prognosis of Patients with Secondary Knee Traumatic Arthritis

Treatment and prognosis of 69 cases of secondary knee traumatic arthritis: according to the investigation, 40 of 69 patients with secondary knee traumatic arthritis were treated with total knee arthroplasty, of which 29 cases were treated with biological fixation of acetabular cup. 11 cases were treated with bone cement acetabular cup fixation, and the other 29 cases were treated with total knee arthroplasty. The HSS scores of biological fixed acetabular cup fixation group, cement acetabular cup fixation group, and total knee arthroplasty group were compared. There was no significant difference among the three groups before and after operation (*P* > 0.05). Comparison within groups, the HSS scores of patients in each group increased pre- and postoperation, and there are statistically significant differences between groups (*P* < 0.05). X-ray examination of 69 patients showed no loosening of prosthesis after operation. The average time between bone grafting and acetabular bony union was 5.05 ± 0.91 months. All results are shown in Table 4.

## 4. Discussion

This study would investigate the risk factors affecting the secondary traumatic arthritis of the knee after the treatment of tibial plateau fractures with internal plate fixation. The structure of the tibial condyle is a spongy bone, which is prone to fracture under the impact of high-energy violence. Clinically, nonoperative treatment and surgical treatment can be selected for tibial plateau fractures. Nonoperative treatment is a conservative treatment. Its indications are incomplete fracture, no displacement, or displacement of the fracture piece < 3 mm. The common treatment methods are plaster fixation, traction treatment, and reduction treatment. Nonsurgical treatment is less traumatic to patients and has a certain scope of application. Foreign scholars believe that nonsurgical treatment is suitable for nondisplaced fractures, and ultraknee splints can be used for external fixation for this type of fracture [16]. Other scholars believe that nonsurgical treatment can be applied to mildly displaced fractures, fracture reduction by manual reduction, and external fixation with an ultraknee splint [17]. Chinese scholars believe that nonsurgical treatment can also be applied to moderately displaced fractures [18].

In order to ensure that patients with tibial fractures can continue a healthy life, a variety of treatment methods have been developed clinically. Among them, the treatment effect of internal plate fixation is better, which has the characteristics of small trauma and high cure rate, and has been widely used in clinical practice. In addition to manual reduction, bone traction and extraknee splint external fixation should also be performed during treatment. When the tibial plateau is damaged by high energy, the articular surface usually collapses. If nonsurgical treatment methods such as traction or external fixation cannot solve the problem of articular surface collapse, it will lead to irreversible articular surface damage. The knee joint is thus affected, and its stability is greatly reduced, which can cause traumatic arthritis of the knee joint for a long time [19]. Surgery needs to meet certain surgical indications. If unstable fractures such as severe displacement of fracture, obvious collapse of articular surface, and ligament injury are found in the examination, surgical treatment must be adopted. The most common treatment is internal plate fixation [20, 21]. Some scholars pointed out that 60 patients with tibial plateau fractures suffered from low energy injury and were treated by internal plate fixation [22]. The patients were followed up for one year, and the results showed that the excellent and good rate of knee joint function recovery was only 85% and 15% of the patients had knee traumatic arthritis [23]. When observing the X-ray films of the patients' knee joints, it was found that different degrees of degeneration could be observed in the patients' knee joints, accounting for 30%. The possible reasons for the degeneration of knee joint function were as follows: firstly, the reduction by surgical treatment may lead to unsatisfactory reduction effect [24]. Secondly, the injured site of the fracture patients healed after treatment, but the weight-bearing line of the knee joint changed compared with that before the injury. Thirdly, because the knee joint was injured and complicated with soft tissue contusion, cartilage hyperplasia and heterotopic ossification appeared after recovery [25].

There are many complications of tibial plateau fractures, including early complications such as infection, vascular injury, soft tissue necrosis, and loss of internal fixation reduction, and late complications such as ankylosis, traumatic arthritis, fracture nonunion, and malunion. The occurrence of complications leads to the difficulty of clinical treatment [26, 27]. The key to the treatment of tibial plateau fracture is how to obtain a knee joint with normal movement, good alignment, painless, and stable. For patients with open tibial plateau fracture, emergency surgical treatment should be taken within 6-8 hours after operation. For patients with closed tibial plateau fracture, if the whole body and soft tissue are in good condition, open reduction and internal fixation should be performed as soon as possible to avoid local tension blisters and even induce osteofascial compartment syndrome, so as not to delay the disease and lose the best time for surgical treatment [28–30]. If the patient has soft tissue injuries, emergency treatment such as drainage and bone traction should be performed first. Open repositioning and internal fixation should be performed after the soft tissue swelling has subsided and the skin texture has returned to normal. Compared with other treatments, the greatest advantage of internal plate fixation is its high stability and very low incidence of displacement [31–33]. Previous clinical studies showed that the operation time, blood loss, and the incidence of postoperative traumatic arthritis in the internal plate fixation group were lower than those in the intramedullary nail fixation group [34]. The postoperative healing rate was higher than that in the intramedullary nail fixation group. However, these methods have fatal shortcomings, which is easy to occur after operation [35, 36]. Therefore, it is very important to find the risk factors that can easily lead to traumatic arthritis after operation.

Combined with the results of this study, tibial plateau fracture is an intra-articular fracture. If the reduction effect is not ideal, it will cause unevenness of the articular surface. Once it exceeds the compensation and regeneration capacity of the knee joint, it will make one side excessive wear and degeneration, resulting in secondary arthritis. Because Schatzker IV is often associated with soft tissue injury and this type of fracture is difficult to achieve anatomical reduction because of more bone fragments, we often classify it as unstable fracture or complex fracture [37, 38]. This study also confirmed that fracture classification and injury mode were the independent risk factors of knee traumatic arthritis after internal plate fixation in the treatment of tibial plateau fracture. Our analysis shows that damage to the soft tissues surrounding the knee joint, or insufficient attention and protection during surgery, can compromise overall movement and coordination mechanisms [39]. In tibial plateau fracture with osteoporosis, the articular surface is prone to collapse and compression, resulting in varying degrees of bone loss. Because of osteoporosis, bone mass is significantly reduced especially in the process of reduction and bone graft. It is difficult to obtain strong fixation [40]. A retrospective analysis of 57 cases of poor reduction of tibial plateau fractures pointed out that strong fixation after anatomical reduction was the key to avoiding or delaying traumatic osteoarthritis [41]. Severe osteoporosis is one of the reasons for the poor effect of fracture reduction. In this group, 69 cases developed secondary knee traumatic arthritis, of which 35 cases were associated with osteoporosis. Our findings were that osteoporosis and the time from injury to operation were independent risk factors, so we considered that osteoporosis was associated with osteoporosis. The main cause of long-term secondary knee traumatic arthritis was poor reduction of fracture. If there was no timely surgical treatment after injury, it might cause continuous damage of soft tissue, increase the difficulty of operation, and lead to traumatic arthritis after operation. After trauma or crush injury, relatively high energy injury can easily lead to joint compression and damage most blood vessels and nerves. And patients with crush injuries are more likely to develop arthritis after operation. This study still has some shortcomings. Firstly, the quality of this study is limited due to the small sample size we included in the study. Secondly, this research is a single-center study, and our findings are subject to some degree of bias. Therefore, our results may differ from those of large-scale multicenter studies from other academic institutes. This research is still clinically significant, and further in-depth investigations will be carried out in the future.

In conclusion, fracture classification, injury mode, osteoporosis, and time from injury to operation are independent risk factors for knee traumatic arthritis in the treatment of tibial plateau fractures with internal plate fixation, incidence of knee trauma.

## Figures and Tables

**Figure 1:** Incidence of secondary knee traumatic arthritis after operation.

**Table 1:** Monofactor analysis of postoperative secondary knee traumatic arthritis.

Monofactor	Control group (*n* = 231)	Research group (*n* = 69)	*t*/*χ*^2^ value	*P* value
Age	55.19 ± 2.31	55.14 ± 2.44	0.155	>0.05
Gender (male/female)	113/118	34/35	0.002	>0.05
Steel plate type				
Combined steel plate	105 (45.45%)	36 (52.17%)	0.967	>0.05
Anatomical plate	81 (35.06%)	21 (30.43%)		
Locking steel plate	45 (19.48%)	12 (17.39%)		
Fracture classification				
I	0	14 (20.29%)	67.188	<0.05
II	23 (9.96%)	15 (21.74%)		
III	115 (49.78%)	33 (47.83%)		
IV	93 (40.26%)	7 (10.14%)		
Mode of injury				
High energy	135 (58.44%)	12 (17.39%)	35.826	<0.05
Low energy	96 (41.56%)	57 (82.61%)		
Osteoporosis	41 (17.75%)	35 (50.72%)	30.542	<0.05
Meniscus injury	114 (49.35%)	27 (39.13%)	2.227	>0.05
Injury of collateral ligament	42 (18.18%)	18 (26.09%)	2.075	>0.05
Cruciate ligament injury	65 (28.14%)	23 (3.33%)	0.691	>0.05
Time from injury to operation				
≤7 d	157 (67.97%)	31 (44.93%)	12.052	<0.05
>7 d	74 (32.03%)	38 (55.07%)		
Time from operation to weight-bearing				
≤6 months	34 (14.72%)	11 (15.94%)	0.062	>0.05
>6 months	197 (85.28%)	58 (84.06%)		
Removal of internal fixation	77 (33.33%)	21 (30.43%)	0.202	>0.05

**Table 2:** Assignment table.

Dependent variable	Assignment
Fracture classification	I, II = 0, II, IV = 1
Mode of injury	Low energy = 0, high energy = 1
Osteoporosis	No = 0, yes = 1
Time from injury to operation	>7d = 0, ≤7d = 1

**Table 3:** Logistic regression analysis of multiple factors affecting knee traumatic arthritis after internal plate fixation for tibial plateau fracture.

Constant	*b*	S. E	Chi-square value	*P* value	OR	95% CI for OR
Fracture classification	0.891	0.145	37.759	<0.05	2.438	1.835-3.239
Mode of injury	1.241	0.352	12.430	<0.05	3.459	1.735-6.896
Osteoporosis	1.692	0.592	8.188	<0.05	5.441	1.705-17.363
Time from injury to operation	-0.245	0.101	5.884	<0.05	0.783	0.642-0.954

**Table 4:** Therapeutic effect and prognosis of patients with secondary knee traumatic arthritis.

Grouping	*N*	HSS scoring		*t* value	*P* value
		Before operation	After operation		
Biological fixed acetabular cup fixation	29	36.53 ± 4.31	90.84 ± 1.55	63.854	<0.05
Cement fixation with acetabular cup fixation	11	36.40 ± 4.56	91.49 ± 2.35	35.617	<0.05
Total knee arthroplasty	29	36.19 ± 4.11	90.18 ± 2.45	60.763	<0.05
*F* value		0.046	1.725		
*P* value		>0.05	>0.05		

## Data Availability

No data were unavailable in this study due to the patients' privacy.
